This article has been retracted.

# Effect of Aerobic Exercise on Liver Tissue in Rats with NAFLD

**DOI:** 10.1155/2022/4165839

**Published:** 2022-09-10

**Authors:** Li Li, Ruichen Liu, Mengfan Niu, Tongxi Zhou

**Affiliations:** ^1^College of Sports and Human Sciences, Harbin Sport University, Harbin, 150008 Heilongjiang, China; ^2^Graduate Faculty, Harbin Sport University, Harbin, 150008 Heilongjiang, China

## Abstract

**Objective:**

To observe the improvement effect of aerobic exercise on liver tissue of rats with NAFLD, explore whether it can reduce NAFLD symptoms without drug dependence, and provide certain data support for the relief of NAFLD by aerobic exercise.

**Methods:**

40 healthful male SD rats have been divided into ordinary diet and high-fat diet. To observe whether the molding is forming after 6 weeks, then divide the rats into control (C), model (M), and exercise (E) group. E group received 8-week aerobic exercise intervention. Serum and liver samples were taken and analyzed after the last intervention.

**Results:**

The morphological of hepatocytes between C and M group becomes different, and the accumulation of fat and inflammatory cells was significant, suggesting that NAFLD symptoms appeared, that is, the model was successfully established. Compared with M group, the morphology of rats in E group was improved in varying degrees. The quantity of ALT, AST, and MDA of rats in M group is increased, and the SOD activity is significantly reduced (*P* < 0.01). However, aerobic exercise intervention changed those result (*P* < 0.01).

**Conclusions:**

Aerobic exercise can relieve oxidative stress damage, lipid peroxidation levels, and chronic inflammatory status in rats with NAFLD, which can reduce NAFLD symptoms without drug dependence, and is expected to become a means of NAFLD treatment.

## 1. Introduction

In recent 25 years, the global population with nonalcoholic fatty liver disease (NAFLD) accounts for more than one-quarter of the total population. In the past, most studies believed that NAFLD is a harmless benign disease, which has nothing to do with cryptogenic cirrhosis. However, with the continuous increase of patients with NAFLD and the deepening of relevant pathological research, researchers have now equated NAFLD, nonalcoholic steatohepatitis (NASH) with the risk of cryptogenic cirrhosis. It is considered that nonalcoholic fatty liver fibrosis and nonalcoholic fatty liver cirrhosis are the downstream effect products of the development of NAFLD and NASH [1].

According to the recent epidemiological survey results at home and abroad, the prevalence and detection rates of NAFLD worldwide are increasing year by year, and the prevalence rate was 6.3~45%. The fluctuation of NAFLD prevalence in China is also parallel to the trend of metabolic related diseases. Moreover, the unique dietary culture tradition also results in the accumulation of body fat, especially visceral fat. In 1995, the proportion of NAFLD in China was only 3.87%. So far, it has increased to nearly 30%, so it has become one of the serious threats affecting of life of Chinese people [2]. Our demand for the inquire about on the pathogenesis of NAFLD and the improvement of clinical drugs has gotten to more and more apparent.

### 1.1. Development Status of NAFLD

Since the discovery of NAFLD, the scientific name of NAFLD has been changed iteratively with the in-depth study of NAFLD. In 1980, Ludwig et al. found that there were significant fatty degeneration, inflammatory infiltration, fibrosis, and focal necrosis in liver biopsy samples from 20 patients. They had no drinking history, and most of them had metabolic diseases such as obesity, diabetes, and gallstones. They named the newly discovered liver disease nonalcoholic steatohepatitis (NASH) [3]. By 2002, follow-up studies found that Nash was only one of the pathological stages of this liver disease, so this liver disease was broadly named nonalcoholic fatty liver disease. By 2020, studies have found that NAFLD and many chronic metabolic diseases are mutually causal. NAFLD is considered to be the closest relationship with metabolic dysfunction. At the same time, studies believe that the part of speech of “nonalcoholic” is derogatory, which has the implied meaning of discriminating against the patient group, and “nonalcoholic” cannot reflect the heterogeneity of various phenotypes of the disease course. Therefore, NAFLD was renamed metabolically associated fatty liver disease (NAFLD) after the consensus reached by the experts of the international fatty liver group [4]. However, due to the low prevalence of NAFLD as a new disease name of NAFLD, NAFLD is still the mainstream scientific name of this liver disease in China, so NAFLD is still used as the title of this liver disease in this paper.

### 1.2. Progress in Cinesiotherapy of NAFLD

The imbalance of dietary structure, the increase of sedentary time, and the lack of physical activity have gradually become the mainstream lifestyle of contemporary social groups. These three characteristics are common inducement factors of NAFLD. The clinical treatment of NAFLD patients generally focuses on adjustment lifestyle, supplemented by drug treatment. The lifestyle adjustment includes improving dietary structure, adjusting work and rest time, and reasonably arranging exercise. For NAFLD patients with obesity, active weight loss through exercise is an effective measure to treat NAFLD. The study found that the degree of body mass reduction is related to the improvement of liver histology. Reducing body mass by 3~5% can improve hepatic steatosis, and reducing body mass by 10% can improve hepatic necrotizing inflammation. For NAFLD patients without obesity (about 3~30%), exercise can still directly improve the liver condition by reducing sedentary time and increasing physical activity time [5, 6].

At present, personalized exercise suggestions for different types of NAFLD patients have not been implemented. However, various studies have different opinions on comparing the effects of various forms of exercise in the treatment of NAFLD. The results of José et al. [7] animal experiments show that 8-week anaerobic exercise has more significant effects on the improvement of glucose tolerance, insulin resistance, and liver fat of hyperlipidemia rats induced by high glucose diet than aerobic exercise and combined exercise (aerobic + anaerobic). The anti-inflammatory effects of the three exercise modes are similar. Among them, aerobic exercise can reduce the appetite of rats. It effectively reduced the food intake of rats but did not reduce their body mass. Still, the improvement of insulin resistance and body mass should benefit from the dual intervention of exercise and diet management. The results of clinical trials showed that three months of aerobic exercise (40% maximum oxygen uptake intensity) could simply improve the level of oxidative stress injury and inflammation in patients with obese NAFLD [5]. So far, many studies on the mechanism of aerobic exercise on NAFLD have been carried out at home and abroad, and many scholars have recognized its effectiveness. Studies at this stage believe that aerobic exercise can treat NAFLD by improving insulin resistance; reducing oxidative stress injury, inflammatory response, and apoptosis; and inducing hepatocyte protective autophagy. It has comprehensive and comprehensive characteristics in the therapeutic effect. Therefore, this study selects medium-intensity aerobic exercise as the form of exercise intervention in this experiment.

To sum up, NAFLD has good exercise sensitivity, and various forms of exercise can be used as nondrug therapy and active recovery means of NAFLD. Exercise not only has the advantages of simplicity, economy, safety, and nontoxic side effects but also has the characteristics of comprehensiveness and comprehensiveness in the treatment effect.

## 2. Methods

Sprague-Dawley male rats (40) were selected for this study, of which 14 were in the ordinary diet group and 26 were in the high-fat diet group. Two rats in each group were killed after 6-week, and liver tissues were taken for hematoxylin-eosin staining observation. The remaining 12 rats in the normal diet group were changed to control group (C), and the high-fat diet group was divided into model group (M) and exercise group (E). E group conducted 8-week exercise intervention with reference to Zhou et al. [8]: 7 d/w, 60 min/t, and 15 m/min (Figure 1). The rats were euthanized at twenty-four hours after the intervention experiment. The serum was obtained and analyzed for alanine aminotransferase (ALT) and aspartate aminotransferase (AST). The liver tissue was taken for HE staining and analyzed for superoxide dismutase (SOD) and malondialdehyde (MDA) analysis. All analyses were performed with SPSS 21.0 (IBM, USA), and *P* < 0.01 was considered statistically significant.

## 3. Results

### 3.1. Observation of Liver Histomorphology after Intervention

After 14-week feeding, comparing the hepatocytes of rats in M group, it was found that the high-fat diet changed the hepatocytes of rats, with obvious fat accumulation and inflammatory cell aggregation. After the intervention, the state of hepatocytes in E group was significantly improved (Figure 2).

### 3.2. Serum Indexes

The levels of ALT and AST in serum of M group were significantly higher than those of C group and E group (*P* < 0.01) (Figure 3 and Table 1).

### 3.3. Liver Tissue Indexes

The levels of SOD and MDA in liver tissue of M group were significantly different from those of C group and E group (*P* < 0.01) (Figure 4 and Table 2).

## 4. Conclusions

Hepatic steatosis is the initial factor in the progression of NAFLD, and oxidative stress and inflammatory response that are closely related to insulin resistance are the physiological and pathological basis of the progression of NAFLD. Due to obesity, overweight, genetic susceptibility, and other reasons, the body produces insulin resistance, leading to liver steatosis, and the excessive accumulation of FFA in liver tissue leads to lipotoxicity, resulting in the damage of liver cells by oxidative stress and endoplasmic reticulum stress until apoptosis [9]. Therefore, this experiment chose to compare the effects of aerobic exercise intervention on NAFLD rats.

The results of this experiment show that after 14 weeks of high-fat diet feeding, the quantity of ALT, AST, and MDA of rats in M group is increased, the SOD activity is significantly reduced. It indirectly indicates that the ROS level of liver tissue of rats in M group has been significantly increased, and the oxidation and antioxidant system in liver tissue of rats has been unbalanced. It is verified that high-fat diet can induce hepatic steatosis and then lead to oxidative stress injury and lipid peroxidation injury. After 8-week exercise, the levels of ALT, AST, SOD, and MDA of rats in E group had significant improvement with M group (*P* < 0.01). It shows that aerobic exercise can improve NAFLD.

Collectively, the aerobic exercise intervention adopted in this study can effectively improve the liver tissue morphology and function of NAFLD model rats and can alleviate the oxidative stress injury, lipid peroxidation level, and chronic inflammation of NAFLD model rats by increasing the SOD activity and reducing the ALT, AST, and MDA content.

## Figures and Tables

**Figure 1:** Experimental design.

**Figure 2:** Liver sections after intervention (×200). Note: (a) C group; (b) M group; (c) E group.

**Figure 3:** Serum indexes. Note: (a) ATL; (b) AST. Compared with C group, ^∗∗^*P* < 0.01; compared with M group, ^##^*P* < 0.01.

**Figure 4:** Liver tissue indexes. Note: (a) SOD; (b) MDA. Compared with C group, ^∗∗^*P* < 0.01; compared with M group, ^##^*P* < 0.01.

**Table 1:** Serum indexes (*x* ± *S*) (*n* = 12).

Indexes group	C group	M group	E group
ALT(U/L)	60.06 ± 2.59	107.48 ± 3.26^∗∗^	87.23 ± 7.45^##^
AST(U/L)	99.91 ± 5.13	138.07 ± 8.67^∗∗^	123.56 ± 6.46^##^

Note: compared with C group, ^∗∗^*P* < 0.01; compared with M group, ^##^*P* < 0.01.

**Table 2:** Liver tissue indexes (*x* ± *S*) (*n* = 12).

Indexes group	C group	M group	E group
SOD (U/mg)	249.40 ± 14.47	127.17 ± 6.69^∗∗^	214.97 ± 7.52^##^
MDA (nmol/mg)	1.62 ± 0.13	6.56 ± 0.15^∗∗^	2.52 ± 0.38^##^

Note: compared with C group, ^∗∗^*P* < 0.01; compared with M group, ^##^*P* < 0.01.

## Data Availability

The data that support the findings of this study are available from the corresponding author upon reasonable request.
